The article "The Effects of Insertion Approach on the Stability of Dental Implants" was published in 2022. Journal: Appl Bionics Biomech.

# The Effects of Insertion Approach on the Stability of Dental Implants

**DOI:** 10.1155/2022/7188240

**Published:** 2022-02-14

**Authors:** Yuan-Yang Hsu, Heng-Li Huang, Lih-Jyh Fuh, Ming-Tzu Tsai, Jui-Ting Hsu

**Affiliations:** ^1^School of Dentistry, College of Dentistry, China Medical University, Taichung 404, Taiwan; ^2^Department of Bioinformatics and Medical Engineering, Asia University, Taichung 413, Taiwan; ^3^Department of Dentistry, China Medical University and Hospital, Taichung 404, Taiwan; ^4^Department of Biomedical Engineering, Hungkuang University, Taichung 433, Taiwan

## Abstract

Dental implant surgery involves the insertion of a dental implant into the alveolar bone; the success of the surgery depends on the initial stability of the implant. The objective of this study was to examine the effects of dental implant insertion approaches in clinical surgery and in accordance with the standards of American Society for Testing and Materials on initial implant stability. Three insertion approaches were used for dental implant placement (Branemark Systems NobelSpeedy Groovy, Nobel Biocare AB, Gothenburg, Sweden) in two types of artificial bone—good bone (GB) and poor bone (PB). The three insertion approaches were as follows: (1) continuous rotation insertion (CRI): using a torque testing machine to continuously screw in an implant to completion and (2 and 3) intermittent rotation insertion (IRI)_90 and IRI_80: using CRI to bury an implant to 90% and 80% of its full length followed by IRI to complete the implantation, respectively. The maximum insertion torque value (ITV), periotest value (PTV), and implant stability quotient (ISQ) were measured and compared. The results indicated that bone quality and insertion approach both affected implant stability. Insertion approaches affected all three implant stability indicators differently in the GB and PB groups (*p* = 0.008). In GB groups, the insertion approach primarily affected ITV, whereas in PB groups, it primarily affected PTV. The effect of the insertion approach was less apparent for ISQ. Overall, in both the GB and PB groups, the implant stability for IRI_80 was greater than that for IRI_90, and the implant stability for IRI_90 was greater than that for CRI. Future *in vitro* studies should adopt an insertion approach that complies with the clinical practice for dental implant surgery. Dentists should adjust the timing for IRI in dental implant surgery to achieve greater initial dental implant stability.

## 1. Introduction

Factors such as caries, periodontal disease, or trauma can cause tooth avulsion or necessitate tooth extraction [1]. If a missing tooth is not replaced by a denture, the resulting gap can affect mastication and pronunciation or even result in alveolar bone resorption [2]. Moreover, the gap can become an aesthetic problem if it is located in the anterior region. Dental implant surgery is one of the treatments to replace missing teeth. A dental implant, which is made of biocompatible titanium, is inserted into the alveolar bone to allow the attachment of osteocytes. After the titanium implant has completely integrated with the alveolar bone, it can act as an abutment for a denture [3]. The success of dental implant surgery is determined by the initial stability of the dental implant; implant mobility must be minimal to avoid interference with osseointegration, a process in which osteocytes gradually grow and calcify on the implant [3–7]. If adequate initial stability is not achieved, nonfunctioning fibrous tissues which are similar to scar tissue will form on the surface of the implant; these tissues can cause osseointegration to fail and greatly increase the risk of implantation failure [8]. Numerous factors can affect initial dental implant stability [9–11], such as bone quality and quantity at the dental implant site, shape and surface treatment of the dental implant, and proficiency of the dentist [9–11].

In clinical practice, a predrill hole must be made at the selected dental implant site with a small-bore drill. The diameter of the drill used is progressively increased until the bore of the hole is only slightly smaller than the diameter of the dental implant. Subsequently, a low-speed handpiece is used to perform continuous rotation insertion (CRI) [12]. However, the dental implant is not typically completely screwed in the alveolar bone in one procedure. Instead, after the majority of the dental implant has entered the hole, the remainder is screwed in through intermittent rotation insertion (IRI) using a manual torque wrench [13]. For example, a dentist may screw in 90% of an implant by using a low-speed handpiece, then complete the remaining 10% of the procedure by using a manual torque wrench. Because the insertion process generates torque, maximum insertion torque is typically chosen as an indicator of initial dental implant stability in clinical and laboratory settings. Within a certain range, high torque indicates a strong force that embeds a dental plant into the bone, resulting in high stability [10, 11, 13]. However, the torque generated by each turn of a manual torque wrench cannot be measured. Moreover, several studies have reported that the prefabricated torque wrench rated torque value can be incorrect, resulting in excessive or insufficient exerted torque [14]. Excessive torque may induce marginal bone loss [15], whereas insufficient torques may cause implant instability [9]. To achieve high stability, other insertion tools have been investigated. For example, the capability of electronic torque wrenches to precisely produce rated torque values after prolonged use was studied [16], or various manual torque wrench designs were compared to determine which produced torque most precisely matches its rated value [17].

Dental implant suppliers typically conform to American Society for Testing and Materials (ASTM) F543 when designing products or conducting *in vitro* studies [18–21]. ASTM F543 specifies that a normal force of 1.14 kg must be exerted on an artificial screw or implant, and the implant must be screwed in at 4 rpm or greater with continuous rotation with a torque testing machine [22]. Some *in vitro* studies have explored the feasibility of using smaller predrill holes to improve implant stability when bone quality is weak [22, 23]. One in vitro study analyzed the effects of implant design and artificial bone quality on maximum insertion torque value (ITV) and implant stability quotient (ISQ) and reported that cortical bone one affected ITV but had a minimal effect on ISQ [24]. Regardless, the experimental settings of these *in vitro* studies did not exactly replicate actual clinical practice of dentists screwing dental implants into the alveolar bone.

Therefore, discrepancies exist between laboratory standards and clinical practices. In a clinical setting, a dental implant is usually screwed in at a higher rotational speed, and a portion of it is inserted through intermittent rotation using a manual torque wrench. Conversely, in a laboratory setting, a dental implant is screwed in entirety through continuous rotation using a torque testing machine. To compare the differences between clinical and laboratory practice, this study devised two insertion approaches: (1) CRI, in which a dental implant was inserted in one step, and (2) beginning with CRI and then finishing with IRI. Furthermore, the effect of bone quality on initial dental implant stability was tested by inserting dental implants into two types of artificial bone that differed in bone quality.

## 2. Materials and Methods

### 2.1. Preparation of the Artificial Bone and Dental Implant Components

Two types of artificial bone (Pacific Research Laboratories, Vashon, Washington, USA) that differed in quality were chosen as good bone (GB) and poor bone (PB) in tests. GB mimicked cancellous bone overlaid by a 2.5 mm thick layer of cortical bone. The imitation cancellous and cortical bones were made of cellular rigid polyurethane material (model 1522-12) with an elastic modulus of 137 MPa and a solid material (model 3401) with an elastic modulus of 16.7 GPa, respectively. PB type mimicked cancellous bone overlaid by a 1.0 mm thick layer of cortical bone, imitated by a cellular rigid polyurethane material (model 1522-09) with an elastic modulus of 12.4 MPa and a solid material (model 3401) with an elastic modulus of 16.7 GPa, respectively (Figure 1). The dental implants (Branemark Systems NobelSpeedy Groovy, Nobel Biocare AB, Gothenburg, Sweden) were of dimensions commonly seen in a clinical setting: 4.0 × 11.5 mm (diameter × length).

### 2.2. Three Insertion Approaches of Dental Implant

To ensure that the dental implants were perpendicularly screwed into the artificial bone specimens, predrill holes were created using a precision drilling machine. Dental implants were then inserted using a torque testing machine. A digital torque meter (TQ-8800, Lutron Electronic Enterprise, Taipei, Taiwan) was used to record torques and torque-rotation curves generated when dental implants were screwed into the GB and PB specimens with each insertion approach. Maximum ITV was used to indicate initial dental implant stability (Figure 2). The three insertion approaches were as follows: (1) CRI: continuous insertion of the dental implant using a torque testing machine. That is, an implant 11.5 mm in length was inserted in its entirety by the torque testing machine without pausing. (2) IRI_90: CRI was used to bury an implant to 90% of its full length (i.e., 10.35 mm); then, IRI was used to finish inserting the implant. (3) IRI_80: CRI was used to bury an implant to 80% of its full length (i.e., 9.2 mm); then, IRI was used to finish inserting in the implant. All three approaches were conducted by applying a normal force of 1.14 kg and rotational speed of 4 rpm. During IRI, insertion was paused for 2 s each time the implant rotated 45°. CRI was applied in accordance with standards for *in vitr*o studies as specified by ASTM F543, whereas IRI_90 and IRI_80 were both designed to accurately simulate clinical dental practices.

### 2.3. Measuring ISQ and PTV of the Dental Implant

After the dental implant was screwed into the artificial bone, two parameters for stability were measured: ISQ and periotest value (PTV) (Figure 3). A special clamping device was required to measure both of these values. ISQ was measured using the Osstell ISQ™ wireless resonance frequency analyzer (Osstell ISQ, Osstell AB, Gothenburg, Sweden), with a smart peg mounted on top of the implant. High ISQ values indicate high implant stability.

PTV was measured using a periotest device (Medizintechnik Gulden, Bensheim, Germany). The implant must first be mounted on an abutment and fixed in place with an abutment screw. The distance and angle of the periotest device to the abutment must remain constant. Low PTV values indicate high implant stability.

### 2.4. Statistical Analysis

Three insertion approaches (CRI, IRI_90, and IRI_80) and two types of bone (GB and PB) were used. Therefore, there were six groups in this study. For each group, five specimens were included. For the experimental results, the ITV, ISQ, and PTV of the six groups were reported as median ± interquartile range (IQR). The Mann–Whitney *U* test was applied to compare ITV, ISQ, and PTV of dental implants between the GB and PB groups. The Kruskal–Wallis test was used to compare ITV, ISQ, and PTV of dental implants among the three insertion approach groups and GB or PB groups. Post hoc pairwise comparisons were conducted using the exact Wilcoxon rank sum test with the Bonferroni adjustment, and the significance level was 0.0167 (=0.05/3). All statistical analyses were conducted using SPSS Version 19 (IBM Corporation, Armonk, NY, USA).

## 3. Results

### 3.1. ITV of the Three Insertion Approaches in Two Quality Types of Bone Specimen

For the effect of bone quality on ITV, results indicated that bone quality significantly affected median ITV for all three groups (CRI, IRI_90, and IRI_80). ITV values of implants in GB were all greater than those in PB (Table 1).

The effect of the insertion approach on ITV was evaluated based on whether the bone was GB or PB. For GB, the ITV of CRI (44.1 ± 7.4 N·cm) was smaller than that of IRI_90 (48.4 ± 5.4 N·cm) and IRI_80 (53.4 ± 3.6 N·cm) by 9.8% (*p* = 0.008) and 21.1% (*p* = 0.008), respectively. Additionally, the median ITV for IRI_80 was greater than that for IRI_90, but the difference was nonsignificant (*p* = 0.151). For PB, none of the three insertion approaches were significantly different (*p* > 0.016).

### 3.2. ISQ and PTV of the Three Insertion Approaches for GB and PB

The results indicated that bone quality significantly affected median ISQ and PTV for CRI, IRI_90, and IRI_80 (*p* = 0.008) and that for GB, ISQ was greater, whereas PTV was lower (Tables 2 and 3).

The effects of the insertion approach on ISQ were evaluated based on whether the bone was GB or PB. For GB, the difference between the ISQ of CRI (70.0 ± 2.0) and that of IRI_90 (69.0 ± 1.5) was nonsignificant (*p* = 0.056). Although ISQs of CRI and IRI_90 were both lower than those of IRI_80 (72.0 ± 1.5), differences were only 2.9% (*p* = 0.016) for CRI and 4.3% (*p* = 0.008) for IRI_90. For PB, the ISQ of CRI (58.0 ± 1.5) was not significantly different from that of IRI_90 (57.0 ± 1.0, *p* = 0.548) or IRI_80 (59.0 ± 1.5, *p* = 0.056). Although the ISQ of IRI_80 was greater than that of IRI_90, the difference was only 3.5% (*p* = 0.016) (Table 2).

The effect of the insertion approach on PTV was evaluated for GB and PB. For GB, differences in the three insertion approaches were nonsignificant (*p* > 0.016). For PB, however, the PTV of CRI (10.7 ± 4.5) was greater than that of IRI_80 (8.3 ± 0.7) by 28.9% (*p* = 0.016), whereas the PTV of IRI_90 (8.5 ± 0.6) was not significantly different than that of either CRI (10.7 ± 4.5, *p* = 0.056) or IRI_80 (8.3 ± 0.7, *p* = 0.151) (Table 3).

## 4. Discussion

A comparison of the literature on clinical dental practices and on product development procedures of dental implant suppliers revealed the differences in implant insertion approaches. Specifically, clinical practice involves the use of a low-speed handpiece to perform CRI and partially bury a dental implant, followed by use of a manual torque wrench for IRI to complete the implantation. By contrast, in laboratory practices conforming to ASTM F543, a torque testing machine is used to perform CRI [23]. The effects of the insertion approach on implant stability are unclear; this study was the first comparing clinical and laboratory dental implant insertion approaches. The results indicated that insertion approaches affect initial dental implant stability, particularly in terms of ITV and PTV, regardless of the bone quality of the dental implant site.

In this study, an experiment was performed on artificial bones because fresh cadaver jawbones were difficult to obtain. Even if a sufficient quantity of cadaver bone was available, bone quality would have been inconsistent. Therefore, this study referenced a previous study [24] and chose artificial bones. Two cortical bone thicknesses and two cancellous bone elastic moduli were adopted to simulate two bone quality levels. According to the literature, poor bone quality can result in implant instability, substantially increasing the risk of implantation failure in long-term follow-ups [25]. Furthermore, because the mandible is of superior bone quality compared with the maxilla and because the anterior region is of superior bone density compared with the posterior region [25], dental implant surgery success rates are highest for the anterior mandible and lowest for the posterior maxillary [26]. In consideration of these factors, experiments were performed for two bone quality levels.

Other than bone quality and location of dental implant site, numerous other factors such as the shape or surface treatment of the implant can affect long-term dental implant surgery success rate [3]. After insertion into the alveolar bone, dental implants achieve long-term stability through osseointegration, which requires minimal implant mobility to avoid interrupting osteocyte growth on the implant surface and the formation of fibrous tissues. Therefore, implant stability is a critical factor affecting implant survival [3, 11]. In one study, postoperative follow-ups on 2641 dental implants were conducted to determine the effect of initial dental implant stability on the success rate of dental implant surgery and the failure rate of low-initial-stability implants was 6.2%; the success rate of high-initial-stability implants was 97.5% [27]. Moreover, Javed and Romanos reviewed the literature between 1979 and 2010 and concluded that initial stability governs the success, or failure, of immediate-loading implants [10]. Clinically, ITV, ISQ, and PTV are the three most common indicators of implant stability [28]. ITV is measured during the insertion of a dental implant into the alveolar bone, and the literature indicates that, within a certain range, high ITV indicates high implant stability and consequently high success rates. However, because ITV can only be measured during the insertion of a dental implant, postoperative follow-up is impossible. By contrast, ISQ and PTV are measured after insertion and therefore are suitable for postoperative long-term follow-up investigating implant stability [28, 29].

Clinically, low-speed handpieces are used to perform CRI of dental implants in dental implant surgeries [12]. However, dental implants are typically not screwed in continuously in full length. Instead, in the normal practice, CRI is used to screw in the majority of an implant, and then, IRI is performed using a manual torque wrench for the final portion [12, 15]. In laboratory in vitro studies, CRI to insert an artificial screw or implant is used in accordance with ASTM F543 [18–21] with a torque testing machine at 4 rpm or above and with a normal force of 1.14 kg [23]. Therefore, this study used three insertion approaches to compare clinical and laboratory practices: CRI, IRI_90, and IRI_80. Moreover, two types of artificial bone, differing in bone quality, were tested. The results revealed that bone quality significantly affected initial dental implant stability (ITV, ISQ, and PTV); for all three insertion approaches, significant differences in ITV, ISQ, and PTV (*p* < 0.05) were observed for bone qualities. Specifically, ITV and ISQ were higher and PTV was lower for implants in GB, supporting the findings of most studies [4, 11].

The effects of insertion approach on implant stability were as follows: for ITV, in GB groups, the ITV value of IRI-based approaches was greater than that of the CRI approach, and the value was positively correlated with the length screwed using IRI. Conversely, in PB groups, the insertion approach did not affect ITV. Basically, the ITV would be affected by the insertion approach in the GB groups. For ISQ, in GB groups, the IRI_80 approach resulted in a somewhat greater ISQ (<5%). However, the ISQ would only be minor affected by the insertion approaches in the PB groups. Overall, the insertion approach only slightly affected ISQ in both GB and PB groups. The insertion approach did not affect PTV for GB, but it did for PB. IRI_80 resulted in a 28.9% decrease in PTV compared with the CRI approach. Overall, the insertion approach affected PTV in PB but not in GB.

The effects of bone quality on implant stability were as follows: bone quality affected implant stability, regardless of the insertion approach; implant stability was consistently higher in GB groups than in PB groups. Therefore, it is difficult to enhance the initial stability by changing insertion approaches in the host bone with poor quality. Thus, two-stage dental implant surgery is advisable. That is, first ensure that the dental implant is free of any occlusal loading for 3–6 months to promote osseointegration before installation of the abutment and crown.

For GB and PB, the insertion approach affected implant stability differently. For GB, ITV was greatest for IRI_80. For PB, PTV was lower (i.e., greater stability) for IRI_80. The insertion approach did not significantly affect ISQ. Clinical and ASTM F543 implant insertion methods did result in a difference in initial dental implant stability. Therefore, dental implant suppliers are advised to take clinical practice into consideration in addition to ASTM F543 during product development. Specifically, clinically typical insertion approaches should also be tested. Dentists are advised to begin IRI earlier in dental implant surgery to achieve greater initial dental implant stability.

This study had the following limitations. First, artificial bones were used because fresh cadaver jawbones are difficult to acquire in sufficient quantities. Although artificial bones had optional elastic moduli and consistent quality, they still differ from biological jawbones in some aspects. For example, they have no blood supply or self-healing ability and thus are only suitable for biomechanical analyses and cannot be used to investigate the biological effects on dental implants. Second, all dental implants used in this study were of the same brand; experiments on dental implants of different shapes or with different surface treatments are necessary. Third, only three initial stability parameters were investigated; other biomechanical parameters such as bone-to-implant contact and marginal bone stress and strain were unaddressed.

## 5. Conclusions

Bone quality and insertion approach both affect implant stability. Regardless of the insertion approach, implant stability was higher in bones with greater strength. The effects of insertion approach on implant stability were more complicated; the approaches affected the three implant stability indicators differently in GB and PB groups. In GB, different insertion approaches had significantly different ITV, whereas in PB, PTV was significantly different. The insertion approach had a smaller effect on ISQ. Overall, implant stability for IRI_80 was greater than that for IRI_90, and the implant stability for IRI_90 was greater than that for CRI.

## Figures and Tables

**Figure 1:** Artificial foam bone and dental implant used in this study: (a) artificial bone consisting of cellular rigid polyurethane foam blocks and an artificial solid shell. Right: good bone, left: poor bone. (b) Dental implant.

**Figure 2:** Measurement of the insertion torque value: (a) entire view; (b) closed view.

**Figure 3:** Measuring the initial stability of dental implant: (a) ISQ and (b) PTV.

**Table 1:** ITV of the three insertion approaches for GB and PB.

Insertion approach	Statistical parameters	ITV (unit: N·cm)		*p* value^+^
		GB	PB	
CRI	Median	44.1^a^	16.7^a^	0.008
	IQR	7.4	4.0	
	Max	46.1	18.8	
	Min	33.7	12.2	

IRI_90	Median	48.4^b^	17.1^a^	0.008
	IQR	5.4	2.3	
	Max	53.7	18.7	
	Min	46.5	15.4	

IRI_80	Median	53.4^b^	21.1^a^	0.008
	IQR	3.6	4.5	
	Max	54.7	22.4	
	Min	48.1	15.7	

	*p* value^∗^	0.005	0.08	

ITV: insertion torque value; GB: good bone; PB: poor bone; CRI: continuous rotation insertion; IRI_90: intermittent rotation insertion for the final 10%; IRI_80: intermittent rotation insertion for the final 20%; IQR: interquartile range; Max: maximum; Min: minimum; ^+^*p* value of the Mann–Whitney *U* test; ^∗^*p* value of the Kruskal–Wallis test. Post hoc pairwise comparisons were conducted using the exact Wilcoxon rank sum test with the Bonferroni adjustment; medians with the same letter (a or b) are not significantly different in the same column.

**Table 2:** ISQ of the three insertion approaches for GB and PB.

Insertion approach	Statistical parameters	ISQ		*p* value^+^
		GB	PB	
CRI	Median	70.0^a^	58.0^ab^	0.008
	IQR	2.0	1.5	
	Max	72.0	59.0	
	Min	69.0	57.0	

IRI_90	Median	69.0^a^	57.0^a^	0.008
	IQR	1.5	1.0	
	Max	70.0	58.0	
	Min	68.0	57.0	

IRI_80	Median	72.0^b^	59.0^b^	0.008
	IQR	1.5	1.5	
	Max	74.0	60.0	
	Min	72.0	58.0	

	*p* value^∗^	0.005	0.022	

ISQ: implant stability quotient; GB: good bone; PB: poor bone; CRI: continuous rotation insertion; IRI_90: intermittent rotation insertion for the final 10%; IRI_80: intermittent rotation insertion for the final 20%; IQR: interquartile range; Max: maximum; Min: minimum; ^+^*p* value of the Mann–Whitney *U* test; ^∗^*p* value of the Kruskal–Wallis test. Post hoc pairwise comparisons were conducted using the exact Wilcoxon rank sum test with the Bonferroni adjustment; medians with the same letter (a or b) were not significantly different in the same column.

**Table 3:** PTV of the three insertion approaches for GB and PB.

Insertion approach	Statistical parameters	PTV		*p* value^+^
		GB	PB	
CRI	Median	3.0^a^	10.7^a^	0.008
	IQR	0.8	4.5	
	Max	3.5	17.3	
	Min	2.5	8.5	

IRI_90	Median	3.0^a^	8.5^ab^	0.008
	IQR	0.5	0.6	
	Max	3.3	9.0	
	Min	2.4	8.2	

IRI_80	Median	2.5^a^	8.3^b^	0.008
	IQR	0.3	0.7	
	Max	2.7	8.5	
	Min	2.3	7.6	

	*p* value^∗^	0.053	0.015	

PTV: periotest value; GB: good bone; PB: poor bone; CRI: continuous rotation insertion; IRI_90: intermittent rotation insertion for the final 10%; IRI_80: intermittent rotation insertion for the final 20%; IQR: interquartile range; Max: maximum; Min: minimum; ^+^*p* value of the Mann–Whitney *U* test; ^∗^*p* value of the Kruskal–Wallis test. Post hoc pairwise comparisons were conducted using the exact Wilcoxon rank sum test with the Bonferroni adjustment; medians with the same letter (a or b) were not significantly different in the same column.

## Data Availability

The data used to support the findings of this study are available from the corresponding author upon request.
